# Cardiac stem cell therapy among Clinics of Uncertain Regulatory Status (COURS): under-regulated, under-observed, incompletely understood

**DOI:** 10.1186/s12967-020-02425-6

**Published:** 2020-07-16

**Authors:** Amanda Lindeman, Carl J. Pepine, Keith L. March

**Affiliations:** 1 University of Florida Center for Regenerative Medicine, 1600 SW Archer Rd, PO Box 100277, Gainesville, FL 32610-0277 USA; 2 Division of Cardiovascular Medicine, University of Florida College of Medicine, Gainesville, FL 32610 USA

**Keywords:** Stem cell, Cell therapy, Heart failure, Adipose stem cell, Cardiovascular disease

## Abstract

**Background:**

Although a large body of information exists relating to cellular therapies, much of this information is either anecdotal or has been obtained from relatively small clinical trials, so that the level of evidence available to direct adoption of therapeutic approaches is quite limited. Despite this, a large number of clinics offer various cellular treatments without having gone through the processes of FDA approval. Florida is considered a “hotspot” of such sites, with a large number of clinics relative to the population.

**Methods:**

To better understand the magnitude and scope of this issue with a specific focus on cardiovascular disease, we surveyed clinics in Florida advertising “cell therapy for heart failure”. We identified only 8 clinics that “treat cardiac conditions, including heart failure.” Data on administration route, cell type used, dose, success rate, cost, and training of persons performing procedures were collected when available, via email, telephone, or website information.

**Results:**

A total of 20,135 patients were identified as treated: 2157 for cardiac conditions. All clinics reported administering cells intravenously, using either adipose- or umbilical-derived sources. Doses ranged from 30 to 150 million cells per treatment. The “success rate” ranged from 65 to 85%, with costs from $6000 to $20,700. Procedures were performed by PAs, MDs, and DOs.

**Conclusion:**

Large numbers of patients (> 10% of all 20,135 patients) have been and presumably are still are being treated for “cardiac conditions.” We conclude that implementation of uniform data collection with an outcome registry, as well as creation of a public database listing FDA-approved cell-based clinical trials, would be useful to patients and the cardiovascular field at large.

## Background

Cell-based therapy is gaining momentum as an increasing number of promising, but preliminary, results are presented. With some positive, yet early results, and potential applications across many disease states, clinicians and patients are eager for cell therapy to be incorporated into “standard treatment.” However, like any new treatment, there are many experimental, regulatory, and practical hurdles before sufficient evidence is gathered for this to occur. Despite the fact that this slow, but crucial process is based on a long-standing public health precedent, many clinicians and patients are not prepared to delay. Related to this, a plethora of direct-to-consumer (DTC) outpatient clinics have opened in the United States offering cell-based therapies with uncertain regulatory status, meaning that the cellular products offered are not provided in the context of an IND or IDE. After discussion with a range of leaders in the field, we have termed these clinics “Clinics of Uncertain Regulatory Status” (COURS), and the treatments offered without IND or IDE as “Treatments of Uncertain Regulatory Status” (TOURS).

One potentially important target for cell-based therapies offered by COURS, which is the focus of this communication, is heart failure and other cardiac conditions. In the US, heart failure has a prevalence of 6.2 million and is anticipated to increase 46% between 2012 and 2030, with a predicted prevalence of > 8 million in 2030. In 2014, there were 1 million new cases in those > 55 years old [1]. After diagnosis, survival rates are ~ 50% at 5 and ~ 10% at 10 years [2] and cost 30.7 billion dollars annually [3]. With such costly morbidity and high rates of mortality, heart failure is a major public health issue. Transplantation is the most effective therapeutic option but has major limitations including high cost, organ shortage, and postoperative complications [4]. Thus, cell-based therapy has emerged as a promising therapeutic option based upon trials in animal models and patients, with some evidence of improved outcomes; however, results vary from trial to trial [5].

Despite an incomplete understanding surrounding cell therapy for heart failure, there are a large number of COURS around the U.S. offering some form of it to patients [6]. This treatment has been represented as a form of medical innovation where the goal is the benefit of an individual patient, and is distinguishable from typical clinical trial approaches, where the goal is scientific evidence that can guide management [7]. Because such medical innovation is not driven by results of well-designed trials, it is generally only intended for exceptional circumstances, however, in the field of cell therapy, this type of innovation appears to have become common. This presents a variety of issues including concern for physical harm to patients, concern for psychological harm by fostering unrealistic expectations, inadequate informed consent, and inconsistent or absent follow-up to assess results or patient outcomes.

Current regulatory involvement by the FDA includes guidance that contradicts claims that these COURS are compliant or exempt from compliance. In 2017 the FDA gave clinics offering cell therapy 3 years of “enforcement discretion”. It was indicated that regulations will be enforced more stringently, but not until November 2020, to give COURS time to learn about FDA regulatory pathways and ensure compliance [8].

Considering the prevalence of COURS and their potential for lack of benefit or even possible harm, there is a clear need for clinical data to better understand the products and procedures being used. Turner and Knoepfler [6] surveyed the field of DTC stem cell therapy, finding 351 businesses offering cell therapy in the U.S. “Hotspot” areas where clinics tend to be clustered included California, Florida, Texas, Colorado, Arizona, and New York. As Florida has the highest density of clinics for its population, we chose Florida to begin data collection.

## Methods

Google searches were conducted using the following phrases: “stem cell therapy Florida”, “stem cell clinics Florida”, “stem cell treatment Florida”, “stem cell for heart Florida”, and “stem cell heart failure treatment Florida”. An initial scan of the first 20 pages of results for each search produced 109 websites appearing to be distinct sites offering cell-based treatment. The sample was further narrowed by visiting each of these websites to ensure it met our sample criteria. With exclusion of broken links, companies that did not perform clinical procedures, clinics operating outside of Florida, and clinics that didn’t actually offer cell-based treatments, the sample was reduced to 76 websites. Then each of these websites were thoroughly perused to determine if treatment for heart failure was mentioned. This resulted in only 8 clinics claiming to treat cardiac conditions; of these, 4 clinics explicitly advertised the treatment on their website and the other 4 did not explicitly list conditions they treated, but confirmed treatment of cardiac conditions via follow-up phone call.

From among this selected group of 8 clinics, we attempted to collect the following data: total number of patients treated, number of patients treated for cardiac conditions, route of administration, type of stem cell, dose, success rate, cost, type of personnel performing procedure, frequency of adverse events, publications, academic affiliation, and their understanding of the status of FDA compliance. Initially, we attempted to find these data on clinic websites. Then, we made phone calls and emails to the clinics to ask any remaining questions. It was not possible to collect some data because of lack of information or refusal to answer.

## Results

A total of 20,135 patients were reported as treated with cellular therapeutics across the Florida clinic sites we surveyed; 2157 of these were treated for “cardiac conditions.” All clinics reported that they employed intravenous administration for cardiac indications. They noted using either adipose (7 clinics) or umbilical-derived (4 clinics) sources, with 3 clinics offering both. The estimated doses administered ranged from 30 million to 1 billion cells per treatment, according to 4 clinics that had the information available. The reported “success rate” ranged from 65 to 85% from the 2 clinics that had these data available. Neither clinic could elaborate on how they defined or measured success. The reported price to patients ranged from $6000 to $20,700 for 7 clinics willing to provide these data. The mean price for therapy utilizing adipose tissue-derived cells was $7742 (6 clinics) while the price for umbilical cord tissue-derived products was $12,162 (4 clinics). The mean price across 7 clinics was $9593, while the median price was $6500. By multiplying the median price by the total number of patients treated for cardiac conditions, we estimate that > 14 million dollars were spent by these patients receiving cell therapy for heart failure or associated cardiac conditions.

Cell harvesting and administration were performed by PAs, MDs, and DOs specializing in surgery, internal medicine, or pain management, with only one clinic reporting presence of a “cardiac specialist” and another clinic reporting presence of a “stem cell scientist.”

Adverse events were reported as none (3 clinics) or described as few (4 clinics): one clinic reported occurrence of flu-like symptoms after cord blood, which was rectified by switching to a Wharton’s jelly product; another clinic simply reported adverse events rates as < 1%; another reported one adverse event related to the injection itself; and one clinic reported 2 cases of “pseudo-sepsis.”

Publications related to their stem cell treatments were reported by 3 of 8 clinics. One clinic reported having a previous partnership with an academic institution, one was “working on” a future academic partnership, and a third had a doctor who is a clinical professor at a local institution. All clinics claimed to either be “in compliance” with FDA regulations or “exempt” from FDA regulations entirely. One clinic stated treatment is legal under “right to try,” another said “stem cells are not drugs and therefore are not under FDA regulations,” another cited their compliance “as indicated by only treating diseases with significant clinical evidence,” another said they “follow FDA procedures for sterility and handling of cells,” another specifically cited “compliance via the same surgical procedure exception of 21 CFR 1271,” and 2 others simply said that they were “compliant,” but provided no further explanation.

The questions presented to the clinics and the questions that were answered are summarized in Table 1.

**Table 1:** Questions answered by each clinic

	Publications	Academic affiliation	View of FDA compliance	Administration	Cell types	Dose	Cost	Personnel performing procedures	Total number of patients	Number of cardiac patients	Success rate	Adverse events
Clinic 1	✓	✓	✓	✓	✓	✓	✓	✓	✓	✓	✓	✓
Clinic 2	✓	✓	✓	✓	✓	✓	✓	✓	✓	✓	✓	✓
Clinic 3	✓	✓	✓	✓	✓		✓	✓	✓	✓		✓
Clinic 4	✓	✓	✓	✓	✓	✓	✓	✓	✓			✓
Clinic 5	✓	✓	✓	✓		✓	✓	✓	✓	✓		✓
Clinic 6	✓	✓	✓	✓	✓	✓	✓	✓	✓			✓
Clinic 7	✓	✓	✓	✓	✓		✓	✓				✓
Clinic 8					✓			✓	✓	✓		

A check mark indicates an answer was provided

## Discussion

The US Food and Drug Administration (FDA) is responsible for regulating cell-based therapy as tissue and tissue products, under the broader category of vaccines, blood, and biologics. The use of bone marrow and umbilical cord blood-derived stem cell preparations has historically been permitted by FDA to treat hematopoietic system disorders, including cancers such as leukemia and other disorders [9]; but most other putative cell therapies currently fall under FDA oversight.

In 2017, FDA released 4 guidance documents providing clarification of regulations, which imply that the large majority of these COURS are not compliant. Following this, the FDA sent “regulatory correspondence” to at least 46 clinics and has pursued legal action against two stem cell clinics [10]. FDA Commissioner Scott Gottlieb, MD, has said the following about this transition [11]:

“We support sound, scientific research and regulation of cell-based regenerative medicine, and the FDA has advanced a comprehensive policy framework to promote the approval of regenerative medicine products. But at the same time, the FDA will continue to take enforcement actions against clinics that abuse the trust of patients and endanger their health with inadequate manufacturing conditions or by purporting to have treatments that are being manufactured and used in ways that make them drugs under the existing law but have not been proven safe or effective for any use.”

### Is cell therapy risky or life changing?

Several publications have detailed adverse aspects related to the unregulated field of cell-based therapy including severe vision loss, infection and even death [12–14]. Unregulated procedures and products create an environment in which severe, yet avoidable, complications can occur. However, there are many hundreds of anecdotal case reports, often provided by the treated individuals by means of video or audio recordings, of therapeutic benefits perceived as significant.

Previous reports highlight “sensationalism” within the field and how COURS use it to recruit patients by advertising sweeping, potentially hyperbolic efficacy claims while minimizing potential risks [15, 16].

COURS offering cell therapy have been known to cite Right to Try (RTT) legislation as a justification for operating outside of the FDA. The Right to Try Act, formally known as the Trickett Wendler, Frank Mongiello, Jordan McLinn, and Matthew Bellina Right to Try Act, was signed in May of 2018 to allow patients meeting certain criteria to be able to access experimental treatments. Eligible patients must have a life-threatening condition, have exhausted approved treatments, and be unable to enroll in a clinical trial as certified by a qualified physician. Eligible investigational drugs must have completed a Phase 1 safety trial, have not already been approved by the FDA for any use, and have an IND application which has been filed with the FDA. With the limited information provided by COURS, it is not possible to determine whether they are truly practicing under this law as it is intended. Heart failure is certainly a life-threatening condition, however, it is not known whether particular COURS ensure that each patient being treated has been certified by a physician to be unable to enroll in a clinical trial and has exhausted current treatment options.

Additionally, it is unclear whether patients are providing reasonable informed consent. Informed consent requires not only a detailed outline of the risks and benefits of the procedure but also a statement on the evidence available, or lack thereof (as is relevant with many cell therapies). Lysaght et al. addressed the legal standpoint that a person can only consent to medical intervention when it is substantiated by a tangible benefit, implying that any treatment without evidence of therapeutic benefit cannot be consented to [17].

An unexpected consequence of receiving these stem cell therapy treatments at COURS is that such treatment often excludes the patient from clinical trials designed to gather scientific evidence. The patient may not be made aware of this outcome. Furthermore, the costs can render patients less able to pay for or have their insurance cover standard-of-care treatments of proven benefit for their heart failure [18]. This not only is detrimental to patients themselves, but in a broader sense, to both the field of cell therapy and society at large. In that regard, the fact that COURS are essentially competing with clinical trials for the same patient population tends to render recruitment for FDA-approved cell therapy clinical trials more difficult.

These issues highlight potential damage COURS can inflict on both individual patients as well as the cell therapy field. Despite these concerns, the large number of “success stories” relayed from patients should not, and cannot, be ignored. A considerable number of clinics advertise patient testimonials on their websites and many claim to have received relief, which, for those with chronic life-altering conditions, can be a major improvement in quality of life. Future regulation can help ensure that patients receiving credible treatment are permitted to continue to do so, while at the same time investigating clinics that may be unsafe. The goal should be to halt procedures that are not pursuing evidence supporting safety and efficacy, while facilitating the study and ultimate provision of therapies and procedures that are based upon sound scientific evidence.

### Recommendations from experts in the field

With 8 million Americans seeking medical advice online every day, Liska et al. emphasized the importance of educating patients to prevent misinformation, maintaining open relationships between patients and their primary care physicians, and formation of a Stem Cells Ethics Consortium [19]. They noted the important role physicians will need to play in assisting their patients in making informed decisions about their healthcare (e.g. “participatory medicine”); they suggested that physicians should at first discourage experimental treatments at locations that are presumed to be COURS, while also taking care not to stigmatize their patients in order to preserve open communication. Should patients decide to exercise their right of bodily autonomy and pursue experimental treatment, physicians should educate patients about the risks and help guide them to reputable sources of treatment.

Others have called for even more involvement from physicians, including combating a perceived “era of misinformation” by challenging sweeping marketing messages provided by COURS. Additionally, they call for involvement of state medical boards to set guidelines for what is and is not appropriate and to sanction members (fines, restrictions, suspensions, and even license revocation) when demonstrating unprofessional conduct [20].

The International Society for Stem Cell Research (ISSCR) created a task force to develop *Guidelines for the Clinical Translation of Stem Cells* [21]. These guidelines offer professional and ethical recommendations for researchers and clinicians involved in administering stem cell-based therapy. They emphasize the importance of peer review of procedure and rationale by experts in the field. They highlight the concept that systematic assessments of cellular products are vital to maintaining patient safety, and recommend that clinicians and researchers take special care during the informed consent process to ensure that patients understand the unique risks of stem cell therapy. The guidelines call on researchers and clinicians to monitor patients, report adverse events, and promote transparency wherever possible. Finally, while the ISSCR guidelines acknowledge the unique circumstances surrounding clinicians treating severely ill patients, they also assert that these clinicians should make a commitment to move to a formal clinical trial after experience with a few patients [21].

Knoepfler proposed that dubious clinics could be identified by a lack of affiliation with academic institutions, few publications, and no investigational new drug (IND) or investigational device exemption (IDE) application [22]. While it cannot be argued that all clinics with these characteristics are by default negligible or unethical, it seems reasonable that patients should be wary of these kinds of clinics.

### Strengths and limitations

This is an initial effort to collect data important to better understand “cell-based therapies in the field”. We observed that despite Florida being the third largest state in population and being identified as a “hotspot” of COURS, it was possible to identify only a small number of locations that actually treated heart failure patients. This suggests that most COURS avoid these high-risk patients. Going forward, we document the need for instruments to uniformly collect these data.

We acknowledge a number of limitations to our study. It is likely that these data underestimate the actual number of clinics in Florida that offer cell therapy for heart failure, since there may be clinics that treat heart failure but do not advertise it. Accordingly, it is not possible to confirm that our sample included all of the providers who treat heart failure in a COURS. Thus, our work should be viewed as the beginning of an effort to better define and assess the use of cell-based therapy for cardiovascular disease. Additionally, we recognize that the lack of information related to patient history, including specific diagnoses concerning the nature of the “heart failure” (e.g., heart failure with reduced vs. preserved ejection fraction) or “cardiac conditions” available from the clinics limits the analysis of our data. This is in part related to the common reliance on patient testimonials rather than objective benchmarks or patient-reported outcomes gathered in a pre-specified manner. Finally, we make no statement on credibility of any clinics presented at this time.

### Recommendations

While reasonable primary goals would be to promote safety and scientific innovation concurrently, it is imperative that steps be taken to ensure these aims are being considered. With these goals in mind, possible recommendations include the following:

First, we recommend movement as quickly as feasible into IDE and IND-based trials, in conjunction with strongly advised participation in outcomes registries, to allow data collection on safety and patient outcomes and, ultimately, evaluation of treatment approaches. We estimate > $14 million have been spent in treatment of heart failure at COURS, in Florida alone, without data collection. If this money had been used to fund clinical trials with uniform data collection, it is likely that selected cardiac indications would be closer to approval for marketing. It is not only imperative that patients shift from COURS to FDA-approved clinical trials, but it is important that data accumulated from FDA-approved clinical trials can be synthesized in such a way that facilitates the progression of the regulatory process.

Second, we advocate standardized protocols for cell processing and administration for COURS as they elect to transition to IDE/IND-based trials, thus becoming Clinics with FDA-Approved Regulatory Status (CARS). Simply collecting data from COURS is not sufficient; these data need to be obtained as uniformly as possibly to permit them to be analyzed collectively. However, this becomes difficult when procedures and products are widely varied. Thus, efforts to arrive at consensus on protocols not only for elements such as cell harvesting and administration, but also for outcome measures and general data collection would minimize this barrier. We suggest that it would be useful to employ a designation for providers who adhere to such standardized protocols, such as a certification or compliance notice.

Lastly, a practical and readily implemented approach should include creation of a user-friendly database available to the public, allowing patients to access a list of cell-based trials with FDA clearance via IDE or IND. This would assist patients in readily locating CARS rather than COURS to best ensure safety and efficacy, as well as encouraging patients to receive experimental therapies along with data collection in a manner that advances the field and ultimately good patient care.

## Conclusion

Large numbers of patients have received cell-based therapies for “cardiac conditions” in settings with uncertain regulatory status, but information about results is limited. Implementation of uniform data collection with an outcome registry and a public database of FDA-approved cell-based clinical trials would be useful to patients and the cardiovascular field.

## Data Availability

All data generated or analyzed during this study are included in this published article.

## Abbreviations

CARS: Clinics with FDA-Approved Regulatory Status
COURS: Clinics of Uncertain Regulatory Status
DTC: Direct-to-consumer
FDA: US Food and Drug Administration
IDE: Investigational device exemption
IND: Investigational new drug
ISSCR: International Society for Stem Cell Research
RTT: Right to Try
TOURS: Treatments of Uncertain Regulatory Status
